This article has been retracted.

# Serum Levels of 25-Hydroxyvitamin D and Functional Outcome among Postmenopausal Women with Hip Fracture

**DOI:** 10.1371/journal.pone.0116375

**Published:** 2015-01-30

**Authors:** Lan-Mei Liu, Shuai-Hua Wang, Chuan-Sheng Fu, Xiang-Zhen Han, Bao-Fu Wei

**Affiliations:** 1 Department of Orthopedics, Linyi People’s Hospital, Linyi, Shandong province, People’s Republic of China; 2 Hand and Foot Surgery Department, Shandong Provincial Hospital, Jinan, Shandong province, People’s Republic of China; Garvan Institute of Medical Research, AUSTRALIA

## Abstract

**Objective:**

The main objective of the current study was to assess the distribution and its prognostic value of serum 25-hydroxyvitamin D (25[OH] D) levels assessed at admission in Chinese postmenopausal women with hip fracture.

**Methods:**

From January 1, 2012 to December 31, 2013, all postmenopausal women with first-ever hip fracture were recruited to participate in the study. Serum 25[OH] D levels were measured at admission. The functional evaluation at the time of discharge was performed by the Barthel Index (BI). The prognostic value of 25[OH] D to predict the functional outcome within discharge was analyzed by logistic regression analysis, after adjusting for the possible confounders.

**Results:**

In our study, 261 patients were included and assessed. In the 76 patients with an unfavorable functional outcome, serum 25(OH) D levels were lower compared with those in patients with a favorable outcome [11.8(IQR, 9.9–16.1)ng/ml; 16.8(IQR, 13.6–21.4)ng/ml, respectively; P<0.0001]. In multivariate analysis, there was an increased risk of unfavorable outcome associated with serum 25(OH) D levels ≤ 20ng/ml (OR 5.24, 95%CI: 3.11–8.15; P<0.0001) after adjusting for possible confounders.

**Conclusions:**

Our data support an association between serum 25[OH] D levels and prognosis in Chinese postmenopausal women with hip fracture.

## Introduction

Vitamin D deficiency is a common condition worldwide. People suffering from vitamin D deficiency are susceptible to osteoporosis and fractures [1]. Postmenopausal women who were vitamin D deficient and had high serum levels of retinol had an eight times higher risk of having osteoporosis [2]. The prevalence of vitamin D deficiency in patients with acute hip fracture has been reported widely in recent years, and the vitamin D nutritional status in such reports is usually evaluated based on serum 25-hydroxyvitamin D (25[OH]D).

Hip fracture is the most severe fragility fracture. It is associated with a significant increase in mortality [3] and morbidity [4]. Survivors of hip fracture are at high risk of permanent disability. Up to 25% of them may require long-term nursing home care, and only 40% fully regain their pre-fracture level of independence [5]. Low serum levels of 25[OH] D occur frequently in patients with hip fractures [6].

Previous study found that low serum levels of 25[OH] D was shown to affect independence in activities of daily living, lower extremity function, and risk of falling after hip fracture [5]. Di et al. [7] suggested that serum 25[OH] D was an independent predictor of functional recovery assessed by Barthel Index score after hip fracture. Currently, no data are available on the role of 25[OH] D in the progression of hip fracture in postmenopausal women. In this study, we therefore evaluated the prognostic value of serum 25[OH] D levels assessed at admission in Chinese postmenopausal women with a hip fracture.

## Patients and Methods

Our study was a post-hoc analysis. It was conducted in Department of Orthopedics of Linyi People’s Hospital, Linyi, China. From January 1, 2012 to December 31, 2013, all postmenopausal women with first-ever hip fracture were recruited to participate in the study. Patients with fracture following a road traffic accident and secondary to tumor or primary hyperparathyroidism were excluded. Patients who were on calcium and vitamin D supplements were also excluded from the study. The study was approved by the ethics committee of the Linyi People’s Hospital. All participants were informed of the study protocol and their written informed consent was obtained, according to the Declaration of Helsinki.

Eleven variables were analyzed in each subject as prognostic factors: age, hip fracture type (cervical or trochanteric), cognitive impairment (Mini-Mental State Examination score, _24/30), neurologic impairment (impairment found at clinical examination because of neurologic diseases, mainly Parkinson’s disease or stroke), infections, time between fracture occurrence and blood collection, number of concomitant diseases, surgical procedure type (arthroplasty or internal fixation), sun exposure, activity level and seasons of admission. Cognitive impairment was assessed with the Mini-Mental State Examination [8]. A score below 24 indicates the presence of a cognitive impairment [9]. Activity level was assessed in minutes per day by the LASA Physical Activity Questionnaire [10]. The functional evaluation at the time of discharge was performed by an experienced physician by using the Barthel Index (BI; original version unchanged) [11]. The BI is considered a reliable disability scale for fracture patients. The items can be divided into a group that is related to self-care (feeding, grooming, bathing, dressing, bowel and bladder care, and toilet use) and a group related to mobility (ambulation, transfers, and stair climbing). The maximal score is 100 if 5-point increments are used, indicating that the patient is fully independent in physical functioning. The lowest score is 0, representing a totally dependent bedridden state. In regard to definition of a primary outcome, cut-off score of 50, 60, 75 and 85 were used in previous studies. In our study, according to our clinical practice, the specific cut-off score for the primary outcome definition was 50. A favorable functional outcome was defined as a BI score of 50 to 100 points, while an unfavorable functional outcome was defined as a BI score of 0 to 50 points.

Blood samples of patients and controls were obtained at 7–8:00 in the next morning of the day of admission. 5mL blood was drawn from cubital *vein* by vacuum collection tubes. After centrifugation, aliquots of the samples were immediately stored at −80°C before assay. Serum calcium, phosphorus, alkaline phosphatase (ALP) and Hs-CRP (High-sensitivity- C-reactive protein) were estimated by standard methods using COBAS INTEGRA 800 (COBAS, Basel, Switzerland) on the day of collection. Serum levels of 25[OH] D were measured using the E601 modular (Roche Diagnostics, Mannheim, Germany) with a calibration range from 3 to 70 ng/ml. The intra-assay coefficient of variation [CV] and inter-assay CV were 4.2–7.1% and 5.2%–9.3%, respectively. The 25[OH] D levels were therefore used to classify the vitamin D status into vitamin D deficiency (<20 ng/ml) and vitamin D insufficiency (20～30 ng/ml) [12].

Results are expressed as percentages for categorical variables and as medians (interquartile ranges, IQRs) for the continuous variables. The Mann-Whitney U test and Chi-square test were used to compare the two groups and the elevation ratios. Correlations among laboratory parameters were analyzed using Spearman’s rank correlation test. The influence of serum 25[OH] D levels on functional outcome was assessed by logistic regression analysis, after adjusting for the possible confounders, ie, age, hip fracture type, cognitive impairment, neurologic impairment, infections, time between fracture occurrence and blood collection, number of concomitant diseases, surgical procedure type, sun exposure, activity level, seasons of admission and other biomarkers. Results were expressed as adjusted OR (odds ratios) with the corresponding 95% CIs (Confidence interval). Receiver operating characteristic curves (ROC) analysis was used to test the overall prognostic accuracy of 25[OH] D and other serum biomarkers and results were reported as area under the curve (AUC). All statistical analysis was performed with SPSS for Windows, version 20.0 (SPSS Inc., Chicago, IL, USA) and STATA 9.2 (Stata Corp, College Station, TX), R version 2.8.1. Statistical significance was defined as p < 0.05.

## Results

### Patient characteristics

In our study, 298 patients were admitted. Twenty-one were excluded because their hip fracture was caused by either major trauma or cancer affecting the bone, 16 were excluded because they died or were transferred to other hospitals. The final sample included 261 patients. The median age of patients included in this study was 68 (IQR, 59–79). Among the patients, 10.7% had a family history of fragility fractures, and 23.0% were found to be using medications for comorbid conditions. The median BI at discharge was 70 (IQR, 40–85). At discharge, 29.1% of patients were classified as poor functional outcome. None of the patients were being treated with either vitamin D or its derivatives. The summary statistics of the study subjects was given in table 1.

**Table 1:** Baseline characteristics of patients with hip fracture and controls.

**Parameters**	**Patients(n = 261)**
Age (years), median(IQR)	68(59–79)
BMI(Kg/m2, IQR)	27.0(24.8–28.5)
Inadequate sun exposure (%)	46.7
Season of blood collection (Winter, %)	39.1
History of falls during the last year, median(IQR)	3(1–4)
Number of concomitant diseases, median(IQR)	2(1–3)
Hip fracture type (%)	
Cervical	52.9
Trochanteri	47.1
Concomitant upper-limb fractures (%)	7.3
Surgical procedure type (%)	
Arthroplasty	49.0
Internal fixation	51.0
MMSE<24 (%)	30.7
Neurologic impairment (%)	19.2
Infection needing antibiotics (%)	11.5
Time between fracture and blood collection(hs) median(IQR)	19.8(12.2–27.3)
Hospital stay(days), median(IQR)	18(10–33)
BI at discharge, median(IQR)	70(40–85)
Activity level(min/day), median(IQR)	125(75–200)
Laboratory findings(IQR)	
Serum calcium (mmol/l)	2.26(2.14–2.43)
Serum phosphate (mmol/l)	1.49(1.11–1.83)
Serum ALP (IU/l)	244(140–339)
Serum Hs-CRP(mg dL^−1^)	0.76(0.32–2.17)
Serum 25(0H) D(ng/ml)	15.2(11.8–19.4)
Vitamin D deficiency, n (%)	78.9

Results are expressed as percentages or as medians (IQR); BMI, body mass index; MMSE, Mini-Mental State Examination score; BI, Barthel Index; Hs-CRP, High-sensitivity- C-reactive protein (BMI); ALP, alkaline phosphatise

### Main Results

The results indicated that the median serum 25[OH] D levels was 15.2(IQR, 11.8–19.4)ng/ml. Almost four-fifths of the patients (78.9%) showed deficient levels of 25(OH) D. When functional evaluation at discharge was performed by BI score, there was a significant positive trend between serum 25(OH) D levels and BI score (r [spearman] = 0.384, P<0.0001, Fig. 1). There was a positive correlation between levels of 25[OH] D and Ca (r = 0.298, P<0.0001). In addition, there was significant, albeit weak, negative correlation between 25[OH] D levels and Hs-CRP(r = −0.169, P = 0.006) and ALP(r = −0.151, P = 0.009). There was no correlation between serum levels of 25[OH] D and other factors (P>0.05). Levels of 25(OH) D were compared based on 4 seasons of blood sampling. Significant seasonal differences in 25(OH) D levels were observed ((analysis of variance [ANOVA]: P = 0.006).

**Figure 1:** Correlation between the serum 25[OH] D levels and Barthel Index (BI).

In the 76 patients with an unfavorable functional outcome, serum 25(OH) D levels were lower compared with those in patients with a favorable outcome [11.8(IQR, 9.9–16.1)ng/ml vs. 16.8(IQR, 13.6–21.4)ng/ml, P<0.0001; Fig. 2]. In the multivariate model, 25(OH) D as a continuous variable was an independent predictor of unfavorable outcome, after adjustment for above possible confounders (OR 0.83, 95%CI: 0.79–0.90; P<0.0001). Further, in our study, we found that an increased risk of unfavorable outcome was associated with serum 25(OH) D levels ≤ 20ng/ml (unjusted OR 9.51, 95%CI: 2.87–31.53; P<0.0001). This relationship was confirmed in the dose-response model. In multivariate analysis, there was an increased risk of unfavorable outcome associated with serum 25(OH) D levels ≤ 20ng/ml (OR 5.24, 95%CI: 3.11–8.15; P<0.0001) after adjusting for possible confounders (table 2). In addition, we found that cognitive impairment, age, Hs-CRP and ALP were associated with functional outcome after hip fracture.

**Figure 2:** Distribution of serum 25[OH] D levels in hip fractures women with unfavorable and favorable functional outcome. All data are medians and in-terquartile ranges (IQR). *P* values refer to Mann-Whitney *U* tests for differences between groups.

**Table 2:** Univariate and multivariate logistic regression analysis for functional outcome.

**Parameter**	**Univariate Analysis**			**Multivariate Analysis ^b^**		
	**OR ^a^**	**95% CI ^a^**	***P***	**OR ^a^**	**95% CI ^a^**	***P***
Predictor						
25[OH] D	0.76	0.62–0.83	< 0.0001	0.83	0.79–0.90	<0.0001
Age	1.12	1.04–1.46	< 0.001	1.07	1.03–1.14	< 0.001
Season of blood collection (Winter)	2.29	1.27–4.87	0.024	1.88	0.98–3.59	0.167
Neurologic impairment	3.05	1.81–5.48	0.037	2.11	0.81–4.36	0.236
Cognitive impairment	1.28	1.10–1.54	0.006	1.16	1.03–1.37	0.009
Hs-CRP	1.23	1.05–1.49	0.005	1.09	1.01–1.34	0.011
ALP	1.16	1.09–1.33	< 0.0001	1.12	1.04–1.30	0.001
Ca	1.78	1.24–2.56	0.015	1.54	0.95–3.02	0.143
Fracture type	3.10	1.01–6.66	0.092	—		
Infections	1.35	0.72–2.54	0.921	—		
Number of concomitant diseases	1.20	0.75–1.95	0.464	—		
Surgical procedure type	1.05	0.68–1.62	0.845	—		
Activity level	1.16	1.01–1.42	0.032	1.07	1.02–1.32	0.047
Sun exposure	1.08	1.02–1.24	0.021	1.03	0.89–1.65	0.351
Time between fracture and collection	0.87	0.61–1.24	0.442	—		
25[OH] D(≤20ng/ml)^c^	9.51	2.87–31.53	< 0.0001	5.24	3.11–8.15	<0.0001

^a^Note that the odds ratio corresponds to a unit increase in the explanatory variable.

^b^In multivariate analysis model, the variables included 25OHD, age, season, neurological impairment, cognitive impairment, hsCRP, ALP, Ca, activity and sun exposure.

^c^Serum levels of 25[OH] D ≤20ng/ml as a variable substitute serum 25[OH] D in multivariate analysis model.

OR, odds ratio; CI, confidence interval; Hs-CRP, High-sensitivity- C-reactive protein; ALP, alkaline phosphatise.

Based on the ROC curve, the optimal cutoff value of serum 25[OH] D levels as a predictor for unfavorable outcome was projected to be 15.5ng/mL, which yielded a sensitivity of 82.9% and a specificity of 74.5%, with the area under the curve at 0.838 (95%CI, 0.772–0.901). With an AUC of 0.838, 25[OH] D showed a significantly greater discriminatory ability as compared with age (AUC, 0.54; 95% CI, 0.45–0.63; *P*<0.0001), Hs-CRP (AUC, 0.58; 95% CI, 0.50–0.66; *p*<0.0001) and ALP (AUC, 0.66; 95%CI, 0.57–0.74, P<0.001). Further, in our study, we found that an increased risk of unfavorable outcome was associated with serum 25[OH] D levels ≤15.5ng/ml (adjusted OR 7.11, 95% CI: 3.43–14.15) after adjusting for above possible confounders.

## Discussion

Several factors were associated with BI score after hip fracture. Negative prognostic roles of cognitive impairment, advanced age, and pressure ulcers have already been reported [7]. Our results strongly suggested that serum 25[OH] D levels were significantly lower in patients with an unfavorable functional outcome compared with those in patients with a favorable, and low serum 25[OH] D level (≤20ng/ml) increased poor functional outcome risk in the postmenopausal women with hip fracture (adjusted odds ratio, 5.24[95% CI, 3.11 to 8.15]). To our knowledge, this study is the first to assess the prognostic value of serum 25[OH] D levels assessed at admission in Chinese postmenopausal women with hip fracture. Similarly, another study reported that low serum 25[OH] D level was a significant determinant of poor quality of life in the seosteoporotic women [13]. In addition, a significant positive correlation was found between the serum levels of 25[OH] D and the BI scores assessed at discharge, which was supported by Di et al [7].

In two large-scale investigations in Beijing and Shanghai, as high as 70% to 90% of the participants had blood 25[OH] D levels below 20ng/mL [14–15]. Interestingly, in our study 78.9% of the patients showed deficient levels of 25[OH] D. Similarly, in another hip fracture group, 76.7% of the subjects had vitamin D deficiency, and in the control group, vitamin D deficiency was seen in 32.3% [16]. In fact, 50% of women presenting hip osteoporotic fractures in the United States had serum vitamin D values lower than 12 ng/ml [17]. Likewise, in Italy, 21.6% of patients with hip fracture had hypovitaminosis D [18]. Bakhtiyarova et al. [19] observed significantly lower 25[OH] D concentrations in elderly Russian individuals with hip fractures in comparison with controls.

Whether the low serum 25[OH] D is just an epiphenomenon to fracture severity or independently contributes to prognosis remains uncertain. Several steps essential for muscle contraction have been shown to be regulated by vitamin D. A loss of muscle mass was associated with disability in the elderly, and people with hip fractures are commonly affected by sarcopenia[20]. Skeletal muscles require vitamin D for structural maintenance and optimal function, with deficiency causing loss of muscle mass, an atrophy of type II muscle fibers, and muscle weakness [5]. Furthermore, Vitamin D deficiency results in an abnormal calcium-phosphorus product leading to diminished mineralization of collagen matrix [21]. Jesudason et al. [22] concluded that rises in bone resorption markers and ALP can be detected in postmenopausal women when the serum 25[OH] D level falls below 60nmol/L. Third, vitamin D deficiency affects bone cells that express the vitamin D receptor, thus contributing to the modulation of bone turnover. Overall, severe vitamin D deficiency may result in weaker bones that in turn cause enhanced fracture risk at multiple sites. Fourth, vitamin D deficiency increases the rate of falls [23], in agreement with recent data showing a significant association between vitamin D receptor gene polymorphisms and falls [24]. In addition, vitamin D status was significantly associated with both fall pattern and choice reaction time, a measurement reflecting neuro-protective mechanisms such as central processing, cognition, and motor response [25]. Lastly, severe vitamin D deficiency may increase the risk of multiple concomitant fractures by affecting bone tissue [26], and secondary hyperparathyroidism found in vitamin D-depleted subjects may contribute to impaired muscle function [27].

Some limitations of this observational study should be considered. Firstly, the sample sizes were small and only 76 binary outcome events found in the analysis adjusted for as many as 15 confounding variables. The samples were number limited, potentially causing the bias of our results. In addition, without serial measurement of the circulating 25[OH] D levels, this study yielded no data regarding when and how long 25[OH] D was decreased in these patients. Another limitation was that 25[OH] D measurements were performed after the fracture and may not accurately reflect pre-fracture exposure. Thirdly, we did not collect data to estimate bone fragility in our patients, such as bone mineral density and prevalence of vertebral fractures, and we did not assess parathyroid hormone serum levels. Fourthly, we did not assess vitamin D receptor, which may affect the functional outcome. Fifthly, the effects of circulating 25[OH] D on long-term clinical outcome were not included in the study protocol. Lastly, our study was a single-department study; however, study diversity is also very important and meaningful. Further studies are needed. These studies need to be large, involve multiple centers, and provide statistical confirmation of the prognostic value of serum 25[OH] D in women with hip fracture.

## Conclusion

In summary, these data support an association between serum 25[OH] D levels and prognosis in Chinese postmenopausal women with hip fracture. We recommend that further studies should be carried out with respect to the mechanism between decreased 25[OH] D levels and poor functional outcome. If it is possible to elucidate this, the prognosis of Chinese postmenopausal women with hip fracture might be improved.
